The article "Construction of Endometrial Carcinoma ceRNA Network and Screening of Key Genes Based on TCGA Database" was retracted in 2023. Reasons: signs of a paper mill; suspected computer-generated content; unreliable results or conclusions; concerns about the data.

# Construction of Endometrial Carcinoma ceRNA Network and Screening of Key Genes Based on TCGA Database

**DOI:** 10.1155/2022/1418232

**Published:** 2022-07-04

**Authors:** Yuchun Song, Ping Chu, Pan Li, Fengling Li

**Affiliations:** Department of Gynecology and Obstetrics, Yantai Affiliated Hospital of Binzhou Medical University, Muping District, Yantai, Shandong 264100, China

## Abstract

**Objective:**

Long noncoding RNA (lncRNA) has received more and more attention in human tumor research. This study is aimed at clarifying the regulatory network of lncRNAs-microRNAs- (miRNAs-) mRNAs and at determining the relevant targets in the development of endometrial cancers.

**Methods:**

Download the miRNA, mRNA, and lncRNA expression profile data of endometrial cancer patients from TCGA; use the “DESeq2” package of R software to identify the differential expression of miRNAs, mRNAs, and lncRNAs; construct a network of ceRNA; and perform gene ontology (GO) and Kyoto Encyclopedia of Gene and Genome (KEGG) pathway enrichment assessment on mRNAs in the network of ceRNA; string and Cytoscape 3.7.2 perform PPI assessment on target genes and TOP 10 hub gene screening; Cytoscape 3.7.2 computer program was employed for constructing the lncRNA-miRNA-TOP10 hub mRNA network diagram to determine the signal axis; StarBase database to verify the Top10 hub mRNA expression; the “survival” package in R computer program was implemented to analyze the survival rate of all genes on the lncRNA-miRNA-Top10 hub mRNA network diagram; RT-qPCR to verify the expression level of genes on the signal axis.

**Results:**

1119 differential mRNAs, 14 differential lncRNAs, and 65 differential miRNAs were screened in TCGA; we constructed a ceRNA regulatory network composed of 5 DELs, 7 DEMs, and 90 DEGs; String combined with Cytoscape to screen out Top10 hub genes, namely: LEFTY1, LIN28A, LHX3, ST8SIA3, CEP55, FBXO32, DCN, ANGPTL1, ADRA1A, and KCNMA1; the StarBase database verification results show that ADRA1A, ANGPTL1, FBXO32, KCNMA1, and DCN are downregulated in endometrial cancer tissues; LEFTY1, LIN28A, LHX3, ST8SIA3, and CEP55 are upregulated in endometrial cancer; the constructed lncRNA-miRNA-hub Top10 mRNA network map identified CTD-2314B22, RP11-89 K21/hsa-miR-143, hsa-miR-424/LEFTY1, LIN28A, LHX3, ST8SIA3, and CEP55 signal axis; survival analysis results show that CTD-2314B22, RP11-89 K21, hsa-miR-96, hsa-miR-211, LHX3, ST8SIA3, and DCN are all related to survival; RT-qPCR results indicate CTD-2314B22, RP11-89 K21, LEFTY1, LIN28A, LHX3, ST8SIA3, and CEP55 are upregulated in endometrial cancer cells, and hsa-miR-143 and hsa-miR-424 are downregulated in endometrial cancer cells.

**Conclusion:**

From the perspective of the lncRNA-miRNA-mRNA network, our study identified CTD-2314B22, RP11-89 K21/hsa-miR-143, hsa-miR-424/LEFTY1, LIN28A, LHX3, ST8SIA3, and CEP55 signal axis, which can present considerably potent biomarkers and therapeutic targets for treating endometrial cancer.

## 1. Introduction

Endometrial cancer is a group of epithelial malignancies occurring in the endometrium. The third most common gynecological malignancy leading to death is endometrial cancer, which seriously affects the health and life quality of patients [1]. Among them, postmenopausal females are the high-risk group of endometrial cancer, but 3-14% of patients are in reproductive age, and the proportion of female patients in reproductive age is annually rising [2, 3]. At the present time, the fundamental treatment for endometrial cancer is surgery in combination with chemotherapy and radiotherapy [4]. However, the surgery may require removing part or the entire uterus, which is very difficult for some women of childbearing ages to accept. Furthermore, chemotherapy drugs are highly toxic and have strong side effects, and some patients even develop drug resistance, which critically impact the mental and physical health of patients. After radiotherapy, side effects for endometrial cancer include radiation cystitis, radiation proctitis, vaginal bleeding, nausea, vomiting, and leukopenia [5, 6]. And the recurrence rate of endometrial cancer in the first 3 years after treatment is as high as 15% [7]. Hence, it is necessary to discover the related targets and molecular mechanisms in the pathogenesis of endometrial cancer in order to discover new therapeutic methods and improve the therapeutic effect of endometrial cancer patients.

By developing high-throughput sequencing technology, through large-scale sequencing of various cancers including endometrial cancer, researchers have found that the majority of cancer types have a notable number of RNA molecules that are abnormally expressed at the transcriptome levels. Recently, more and more studies have concentrated on long noncoding RNAs (lncRNAs) [8, 9], which perform an important task in different cellular processes, especially in tumor cells [10]. lncRNAs are transcripts with over 200 nucleotides in length, which are capable of regulating DNA methylation, remodeling of chromatin, and modification of histone, and are miRNAs precursors [11]. lncRNAs can bind to transcription factors to regulate target genes or bind to target sites of microRNA effector complexes, resulting in their loss of regulatory function, or bind to regulatory proteins and jointly participate in the formation of ribonucleoprotein complexes, or recruit DNA-targeted chromatin-modifying complexes, or are directly involved in the regulation and processing of their target mRNAs, through translational repression, splice and splicing, or degradation [12]. miRNAs are single-stranded small RNAs with a size of about 21-23 bases, which could inhibit posttranscriptional gene expression by specifically binding to target messenger ribonucleic acid (mRNA) and play an important role in regulating gene expression and cell cycle [13]. When miRNA acts, it could bind completely to the target gene, and its mode of action and function is very similar to that of siRNA, and finally cleaves mRNA, which is common in plants. It also could be not completely complementary to the target gene when it acts, thereby preventing translation without affecting the stability of mRNA. This is the most discovered mode of action, and it is common in animals. In addition, it has the above two modes of action in the same time [14].

Salmena et al. in 2011 first presented the theory of competitive endogenous RNA (ceRNAs) and found that all types of RNA could be targets of miRNAs, and any target could competitively interact with its miRNAs through the same miRNA reaction element [15]. Recent studies have found that lncRNAs may have the function of ceRNAs and can compete with miRNAs for binding to mRNAs [16]. Subsequent studies on HOTAIR and H19 have also confirmed that ceRNAs may be potential therapeutic targets for cancer [17, 18]. Currently, various explorations have demonstrated that lncRNA NEAT1 boosts the proliferation, migration, and invasion of endometrial cancer cells through the regulation ofmiR-144-3p/EZH2 axis [19]. lncRNA H19 is able to regulate the expression of the relevant target gene HOXA10 in endometrial cancer by competing with miR-612, so that it could promote cancer cell proliferation in the development of endometrial cancer [20]. Although several lncRNA-miRNA-mRNA signaling axes that took part in the pathogenesis of endometrial cancer have been identified, there is still a need for a more comprehensive assessment of the lncRNA-miRNA-mRNA regulatory network and to identify potent targets in endometrial cancer.

Herein, the expression profile information related to endometrial cancer from TCGA was downloaded, screened the differential genes, and created the lncRNA/miRNA/mRNA regulatory network for clarifying the relationship between differentially expressed lncRNA, miRNAs, and mRNAs. The regulatory networks of CTD-2314B22, RP11-89 K21/hsa-miR-143, hsa-miR-424/LEFTY1, LIN28A, LHX3, ST8SIA3, and CEP55 were preliminarily identified, which can present novel perspectives toward the pathogenesis of endometrial cancer.

## 2. Materials and Methods

### 2.1. Dataset Download and Differential Gene Screening

We obtained RNA sequencing data from TCGA. The mRNA and lncRNA sequencing data were obtained from 35 cases of endometrial carcinoma and 553 cases of normal tissue, and miRNA sequencing data from 546 cases of endometrial carcinoma and 33 cases of normal tissue. Employing the “DESeq2” package in the R language, set *P* < 0.01 and ∣log2FC | >3 to obtain differentially expressed lncRNAs (DELs), miRNAs (DEMs), and differentially expressed genes (DEGs) between normal tissues and endometrial cancer tissues, and heatmaps and volcano plots were drawn implementing the “ggplot” and “pheatmap” packages on the R platform, respectively.

### 2.2. Estimation of Target Genes and lncRNAs of DEMs

DIANA-microT (http://www.microrna.gr/microT), miRanda (http://www.microrna.org/microrna/home.d), PicTar (http://www.pictar.org/), and TargetScan (http://www.targetscan.org/) were used for the estimation of miRNA target genes [21], and the overlapping genes of predicted target genes of DEGs and DEMs screened by sequencing data were used as research objects. The database PITA and miRanda (http://genie.weizmann.ac.il/pubs/mir07/mir07_dyn_data.html) were employed for analyzing the interaction between lncRNAs and miRNAs, and the overlapping lncRNAs of DELs and DEMs targeting lncRNAs screened by sequencing data were used as research object for subsequent ceRNA network construction.

### 2.3. Construction of ceRNA Network

On the basis of the ceRNA theory, lncRNAs are able to act as endogenous “sponges” for regulating mRNA expression by downregulating miRNAs. Therefore, mRNAs or lncRNAs with an inverse relationship with miRNAs were selected for constructing a lncRNA-miRNA-mRNA ceRNA network. The visualization of ceRNA networks was carried out by implementing the Cytoscape computer program (version 2.7.2).

### 2.4. Target Gene Functional Enrichment Analysis

GO database is divided into three sections, namely, molecular function (MF), cellular component (CC), and biological process (BP). The database of KEGG allows us to obtain information about the behaviors of genes in diverse pathways in the body. In this study, ClusterProfiler software package of R language was employed for GO and KEGG enrichment assessment of mRNAs in the network of ceRNA, and the screening criterion was *P* < 0.05.

### 2.5. PPI Analysis and Hub Gene Screening of Target Genes

Protein-protein interactions of target genes were analyzed using String (https://string-db) database and subsequently imported the exported “string interactions” file into Cytoscape computer program for visualizing and constructing a network diagram, and the cytohHubba plug-in of Cytoscape computer program was employed for screening the Top10 genes in the network map.

### 2.6. Drawing of lncRNA-miRNA-Top 10 Hub Gene Network Map

The outcomes were imported into Cytoscape software, and the lncRNA-miRNA-Top 10 hub gene network map was constructed using the merge function of the software.

### 2.7. Verification of mRNA Expression

StarBase (http://starbase.sysu.edu.cn/) is an open-source platform to scrutinize the interaction between genes and for the verification of mRNA expression. In this study, the StarBase database was applied for verifying the expression levels of the Top 10 hub genes. *P* < 0.05 was regarded statistically meaningful.

### 2.8. Survival Analysis

The prognostic value of genes was analyzed using Kaplan-Meier (http://www.kmplot.com). To assess the overall survival (OS) in cases suffering from endometrial cancer, the patients were categorized into two groups based on median (high vs. low) gene expression and then validated their Kaplan-Meier survival curve. 95% confidence intervals (CIs) and hazard ratios (HRs) were measured to assess the relationship between genes and survival.

### 2.9. Experimental Verification

#### 2.9.1. Cell Culture

Human endometrial epithelial cells (hEEC) and human endometrial cancer cell lines (Ishlkawa, AN3CA, and HEC-1A) were acquired from the Chinese Academy of Sciences (Shanghai) Cell Bank. The cells were cultivated in Duchenne's altered eagle milieu supplied with 10% fetal bovine serum (Gibco), and the cells were cultivated in a 5% CO_2_ incubator (Adolf Kuhner AG) at 37°C.

#### 2.9.2. The Expression Levels of Genes on CTD-2314B22, RP11-89 K21/Hsa-miR-143, Hsa-miR-424/LEFTY1, LIN28A, LHX3, ST8SIA3, and CEP55 Signaling Axis Were Verified by qRT-PCR

The extraction of total RNA was achieved by employing TRIzol (Invitrogen Company) reagent. Total RNA was reversely transcribed into cDNA according to the PrimeScript RT reagent Kit, and qRT-PCR was executed on the synthesized cDNA using the kit of Fast SYBR Green PCR (Biosharp, Inc.) and ABI PRISM 7300 RT-PCR system (ABI, Inc., USA), and each well was set up with 3 replicates. U6 was employed as an internal reference for miRNA and GAPDH was employed as an internal reference for other genes. Relative quantitative method (2^-△△^CT) was implemented for calculating the relative expression levels of each gene. Each assessment was repeated three times.  Table 1 demonstrates the primer sequences.

### 2.10. Statistical Processing

Data were analyzed using SPSS17.0 statistical computer program (IBM). GraphPad Prism 5.0 was implemented for data processing. The nonparametric Mann–Whitney *U* examination was employed for comparing the two groups, and the Kruskal-Wallis test was applied for comparing more than two groups. *P* < 0.05 illustrated significant discrepancy.

## 3. Results

### 3.1. Screening of DELs, DEMs, and DEGs in Endometrial Cancer

The endometrial cancer-related lncRNA, mRNA, and miRNA data were analyzed from the database of TCGA, and the selection benchmarks of ∣log2FC | >3, *P* < 0.01 were set, and 14 differential lncRNAs were acquired, of which 11 were upregulated and 3 were downregulated (Figure 1), 65 differential miRNAs were achieved, of which 51 were upregulated and 14 were downregulated (Figure 2); and 1119 differential mRNAs were obtained, of which 767 were upregulated and 352 were downregulated (Figure 3).

### 3.2. Determination of Target Genes and lncRNAs of miRNAs and Construction of ceRNA Network

To further comprehend the function of DELs, the ceRNA regulatory network of endometrial carcinoma was established. According to the ceRNA theory, miRNAs were used as the connection point, namely, the interaction pairs of miRNA-mRNA and miRNA-lncRNA, the upregulated miRNA was accompanied by downregulated lncRNAs and mRNAs; and the downregulated miRNA was accompanied by upregulated lncRNAs and mRNAs, the network of lncRNA-miRNA-mRNA ceRNA was created, and a visual network was constructed employing Cytoscape computer program. Further, 13 lncRNA-miRNA regulatory pairs were identified with negative regulatory relationships through the database, including interactions between 7 DEMs and 5 DELs. After identifying lncRNA-miRNA pairs, the target mRNAs of 7 miRNAs were predicted using the DIANA, miRanda, TargetScan, and PicTar databank. A total of 293 genes were achieved from the intersection of the target mRNA of miRNA and the DEGs screened by sequencing. The genes with negative regulation of miRNA were selected, and 90 target genes were finally determined for follow-up research. Finally, we constructed a ceRNA regulatory network consisting of 5 DELs, 7 DEMs, and 90 DEGs (Figure 4).

### 3.3. GO and KEGG Enrichment Evaluation of Target Genes

GO assessment and KEGG enrichment examination were exerted on genes using clusterProfiler of R language. The results of GO assessment illustrated that genes were not enriched in MF and CC, and BP was predominantly enriched in muscle system process, regulation of transmembrane receptor protein serine/threonine kinase signaling pathway, and regulation of cellular response to growth factor stimulus and muscle contraction; the outcomes of KEGG assessment illustrated that genes were substantially enriched in signaling pathways including salivary secretion, vascular smooth muscle contraction, cGMP-PKG signaling pathway, calcium signaling pathway, and renin secretion (Figure 5).

### 3.4. PPI Network Assessment and Top10 Hub Gene Screening

For meticulous exploration of DEGs in the ceRNA network, PPI network assessment was executed by employing the STRING database and Cytoscape3.7.2 software. There were 53 nodes and 42 edges in the network of PPI diagram. The Top10 Hub genes screened by the cytohHubba plug-in were LEFTY1, LIN28A, LHX3, ST8SIA3, CEP55, FBXO32, DCN, ANGPTL1, ADRA1A, and KCNMA1 (Figure 6).

### 3.5. Top10 Hub Gene Expression Verification

The expression levels of Top10 hub gene were verified by StarBase database. The results showed that ADRA1A, ANGPTL1, FBXO32, KCNMA1, and DCN were downregulated in endometrial carcinoma tissues; LEFTY1, LIN28A, LHX3, ST8SIA3, and CEP55 were upregulated in endometrial carcinoma tissues; and the upregulation trend of LIN28A, LHX3, and ST8SIA3 was relatively small (Figure 7).

### 3.6. Construction of lncRNA-miRNA-TOP10 Hub Gene Network Diagram

We drew the lncRNA-miRNA-Top10 hub gene network diagram, from which we can see that lncRNA RP11-366F6 is able to regulate hsa-miR-143, and hsa-miR-143 further regulates LEFTY1 and LIN28A; lncRNA CTD-2314B22 is capable of regulating hsa-miR-143 and hsa-miR-424 and further regulate downstream LEFTY1, LIN28A, LHX3, ST8SIA3, and CEP55 genes; lncRNA FRMD6-AS2 can regulate hsa-miR-96, hsa-miR-182, and hsa-miR-211 and further regulate downstream FBXO32, DCN, ANGPTL1, ADRA1A, and KCNMA1 genes; RP11-89 K21 can regulate hsa-miR-143 and hsa-miR-424 and then regulate downstream LEFTY1, LIN28A, LHX3, ST8SIA3, and CEP55. Among them, CTD-2314B22 and RP11-89 K21 are capable of simultaneous regulating the hsa-miR-143 and hsa-miR-424 and the downstream LEFTY1, LIN28A, LHX3, ST8SIA3, and CEP55 genes. Therefore, this study intends to further verify the levels of expression for these genes through experiments (Figure 8).

### 3.7. Survival Assessment

The prognostic value of all genes involved in the lncRNA-miRNA-Top10 hub gene subnetwork diagram was investigated using Kaplan-Meier. According to the results, we found that CTD-2314B22, RP11-89 K21, HSA-Mir-96, HSA-Mir-211, LHX3, ST8SIA3, and DCN genes were all associated with survival, and the gene expression level was closely correlated with the overall rate of survival for endometrial cancer patients (*P* < 0.05) (Figure 9).The low expression of CTD-2314B22, HSA-Mir-96, HSA-Mir-211, LHX3, ST8SIA3, or DCN gene was closely correlated with the higher overall rate of survival for endometrial cancer patients. And the high expression of RP11-89 K21 was closely correlated with the higher overall rate of survival for endometrial cancer patients.

### 3.8. Expression Level Was Verified by PT-qPCR

Expression levels of CTD-2314B22, RP11-89 K21, LEFTY1, LIN28A, LHX3, ST8SIA3, CEP55, hsa-miR-143, and hsa-miR-424 are in human normal endometrial epithelial cells and human endometrial carcinoma epithelial cells. The results illustrated that CTD-2314B22, RP11-89 K21, LEFTY1, LIN28A, LHX3, ST8SIA3, and CEP55 were all upregulated to varying degrees in endometrial cancer cells, and hsa-miR-143 and hsa-miR-424 were downregulated to varying degrees in endometrial cancer cells (Figure 10).

## 4. Discussion

Recently published investigations have shown that lncRNAs participate in the pathogenesis of many cancers, comprising endometrial cancer. Sun et al. [22, 23] determined 5 lncRNAs (RP11-229P13.20, RP11-275I14.4, VIM-AS1, FLJ27354, and CTB-51 J22.1) that were substantially associated with tumor development and prognosis in endometrial cancer. These lncRNAs provide an independent prognostic predictor. After three or five years, the survival rates of UCEC patients in a predicted high-risk population groups were 80.9% and 68.1%, respectively, while the corresponding ratio for the predicted low-risk group was both 93.9%. Similar research illustrated that lncRNA HOTAIR regulates the metastasis of estrogen-induced endometrial cancer by means of the miR-646/NPM1 axis [24].

Various investigations have illuminated that ceRNAs perform an essential task in the occurrence and advancement of tumors. Because lncRNA is composed of Introns and other segments, the length can reach several thousand nucleotide, which provides a good material basis for the adsorption and binding of a large number of miRNAs. lncRNA can compete to occupy a large number of miRNAs in the cell and then buffer or reduce their ability to interfere with the protein encoded by the mRNA of the target gene like a sponge. These constitute lncRNA-miRNA-mRNA signaling axis [23]. According the ceRNA theory, a ceRNA network was created, which presented helpful clues for next investigations. Regarding the DEGs in the network of ceRNA, GO and KEGG enrichment assessments were conducted, and the findings revealed that DEG genes were enriched in salivary fluctuation, vascular smooth muscle contraction, signaling pathway of cGMP-PKG, calcium signaling pathway, and Renin signaling pathway. Besides, for DEGs in ceRNA network, a network of PPI was created and screened Top10 hub genes, comprising LEFTY1, LIN28A, LHX3, ST8SIA3, CEP55, FBXO32, DCN, ANGPTL1, ADRA1A, and KCNMA1. Lefty-1 can inhibit epithelial–mesenchymal transition and renal interstitial fibrosis by restraining the TGF-*β*/Smad pathway [25]. It has been demonstrated that overexpression of LIN28A boosts the invasion and proliferation of colon cancer cells [26, 27]; overexpression of LHX3 boosts the migration and invasion of tumor cells [28]. The overexpression of ST8SIA3 increases cell proliferation, migration, clone formation, and tumor growth of A2B5+ cells from human glioblastoma in vitro [29]. Notable expression of CEP55 is capable of promoting the proliferation and clone formation of gastric cancer cells [30]. FBXO32 is capable of promoting the apoptosis of ovarian cancer cells and inhibit the growth of cancer cells [31]. Considerable expression of DCN is capable of inhibiting the proliferation of Ishikawa cells in endometrial carcinoma [32]. The ANGPTL1 can inhibit vascular invasion, metastasis, tumor thrombosis, and poor prognosis of hepatocellular carcinoma [33]. ADRA1A was upregulated in peripheral blood of uterine cancer patients, and its expression was related to FIGO stage and lymph node metastasis status [34]. KCNMA1 can augment the proliferation of prostate cancer cells [35], and the above studies indicate that most genes are closely related to cancer. Then, StarBase database was employed to confirm the expression levels of Top10 hub mRNA and found that ADRA1A, ANGPTL1, FBXO32, KCNMA1, and DCN were downregulated in endometrial carcinoma tissues; LEFTY1, LIN28A, LHX3, ST8SIA3, and CEP55 were upregulated in endometrial carcinoma tissues. The constructed lncRNA-miRNA-Top10 hub gene network diagram showed that lncRNA RP11-366F6 regulated hsa-miR-143, and hsa-miR-143 further regulated LEFTY1 and LIN28A; lncRNA CTD-2314B22 regulated hsa-miR-143 and hsa-miR-424, further regulated downstream LEFTY1, LIN28A, LHX3, ST8SIA3, and CEP55 genes; lncRNA FRMD6-AS2 regulated hsa-miR-96, hsa-miR-182, and hsa-miR-211 and further regulated downstream FBXO32, DCN, ANGPTL1, ADRA1A, and KCNMA1 genes; RP11-89 K21 regulated hsa-miR-143 and hsa-miR-424 further regulated downstream LEFTY1, LIN28A, LHX3, ST8SIA3, and CEP55, among which CTD-2314B22 and RP11-89 K21 can simultaneously regulate hsa-miR-143 and hsa-miR-424 and downstream LEFTY1, LIN28A, LHX3, ST8SIA3, and CEP55 genes. It has been illustrated that the expression of CTD-2314B22 in endometrial carcinoma is superior to that in normal tissues [36]; lncRNA FRMD6-AS2 can impede the growth of endometrial cancer cells by increasing FRMD6 in endometrial cancer cells [37]; hsa-miR-143 is able to impede the adhesion, migration, and epithelial-mesenchymal transformation of renal clear cell carcinoma cells and thus play a tumor suppressive effect [38]; miR-424 can be used as a tumor repressor miRNA, which can inhibit migration, invasion, and epithelialization of endometrial cancer cells by targeting regulation of E2F6 gene [39]. For an independent risk factor for prognosis, the high expression of miR-96 suggested that poorer pathological grade and FIGO stage, more myometrial invasion and lymph node metastasis, and poorer 5-year survival rate [40]. miR-182 can promote the proliferation of endometrial cancer cells and inhibit apoptosis through hindering the expression of Foxo1 [41], the above genes have been explained to be relevant to cancer, and these studies further demonstrate the reliability of our bioinformatics analysis. Survival analysis showed that CTD-2314B22, RP11-89 K21, hsa-miR-96, hsa-miR-211, LHX3, ST8SIA3, and DCN were all associated with survival. Next, this study verified the expression levels of genes on CTD-2314B22, RP11-89 K21/hsa-miR-143, hsa-miR-424/LEFTY1, LIN28A, LHX3, ST8SIA3, and CEP55 signaling axis by experiments. Next, this study verified the expression levels of genes on CTD-2314B22, RP11-89 K21/hsa-miR-143, hsa-miR-424/LEFTY1, LIN28A, LHX3, ST8SIA3, and CEP55 signaling axis by experiments. RT-qPCR results showed that CTD-2314B22, RP11-89 K21, LEFTY1, LIN28A, LHX3, ST8SIA3, and CEP55 were all upregulated in endometrial cancer cells, and hsa-miR-143 and hsa-miR-424 were downregulated in endometrial cancer cells.

Briefly, through bioinformatics analysis, we constructed ceRNA network and conducted in-depth analysis on this basis and finally identified CTD-2314B22, RP11-89 K21/hsa-miR-143, hsa-miR-424/LEFTY1, LIN28A, LHX3, ST8SIA3, and CEP55 signaling axis, and the expression of genes on the signaling axis was verified by experiments. The present exploration presents a novel perspective toward the strategy of endometrial cancer, and further studies on the targets and interactions on the signal axis should be carried out in the future.

## Figures and Tables

**Figure 1:** Heat map and volcano map of differential lncRNA identification.

**Figure 2:** Heat map and volcano map of differential miRNA identification.

**Figure 3:** Heat map and volcano map of differential mRNA identification.

**Figure 4:** lncRNA-miRNA-mRNA ceRNA network diagram.

**Figure 5:** GO and KEGG enrichment assessment results of target genes.

**Figure 6:** PPI network and TOP10 hub gene screening. Note: the genes marked in red in the figure are TOP10 hub genes.

**Figure 7:** Expression level results of top10 hub genes were verified using the StarBase database.

**Figure 8:** lncRNA-miRNA-TOP10hub gene network diagram.

**Figure 9:** Survival analysis results.

**Figure 10:** Validation of relative expression levels of genes by RT-qPCR. Note: ∗ indicated *P* < 0.05; ∗∗ indicated *P* < 0.01 vs. hEEC.

**Table 1:** Primer sequence.

Gene	Sense primer	Antisense primer
LEFTY1	CCCAAGCTTGCCATGCCATTCCTGTGGCTCTGC	CGAATTCCTACTTATCGTCGTCATCCTTGTAATCTGGCTGCAGCCTCCTGGGTAT
LIN28A	TTGTCTTCTACCCTGCCCTCT	GAACAAGGGATGGAGGGTTTT
LHX3	ACGGACCCAGTTCTGACCTA	TGGTCTACCTCATCCAGCCA
ST8SIA3	CAAGAACTGAGGAGCACC	TTTCCAACCTTCTACATTGTG
CEP55	TTGGAACAACAGATGCAGGC	GAGTGCAGCAGTGGGACTTT
Hsa-miR-143	UGAGAUGAAGCACUGUAGCUC	GAGCUACAGUGCUUCAUCUCA
Hsa-miR-424	CAGCAGCAATTCATGT	TGGTGTCGTGGAGTCG
CTD-2314B22	AGGCAAGAUGCUGGCAUAGCU	AGCUAUGCCAGCAUCUUGCCU
RP11-89 K21	UAAGGCACGCGGUGAAUGCC	GGCAUUCACCGCGUGCCUUA
U6	CTCGCTTCGGCAGCACA	AACGCTTCACGAATTTGCGT
GAPDH	GAAAGCCTGCCGGTGACTA	AGGGATCTCGCTCCTGGAAG

## Data Availability

The labeled dataset used to support the findings of this study are available from the corresponding author upon request.
